This article has been retracted.

# Breakdancing Movement Based on Image Recognition Promotes Preschool Children's Executive Function and Intervention Plan

**DOI:** 10.1155/2022/1991138

**Published:** 2022-03-07

**Authors:** Feng Tai, Ye Zhang, Yaoxiang Yu, Shijie Zhou, Bo Tan, Chengdong Zhu, Lele Fang, Qiaolin Yu

**Affiliations:** ^1^School of Physical Education, Liaoning Normal University, Dalian 116029, Liaoning, China; ^2^College of Leisure and Social Sports, Capital University of Physical Education and Sports, Beijing, 100088 Beijing, China; ^3^Sports Artificial Intelligence Research Institute, Capital University of Physical Education and Sports, Beijing, 100088 Beijing, China; ^4^School of Psychology, Liaoning Normal University, Dalian, 116029 Liaoning, China; ^5^School of Music, Liaoning Normal University, Dalian 116029, Liaoning, China

## Abstract

With the continuous development of science and technology, people can apply more and more technology to the cultivation of children's abilities. In the process of cultivating children's ability, the most fancy is the study of executive function, and this is the research topic of this article. In the past, training methods such as music, mindfulness, and exercise have been used in the study of children's executive abilities to promote the development of preschool children's executive functions. While various approaches have had some effect, researchers have been exploring more comprehensive approaches to effective training. This article is aimed at studying how to use image recognition technology to conduct an intervention analysis of breakdancing in promoting the executive function of preschool children. For this reason, this paper proposes image recognition technology based on deep learning neural network and conducts research, analysis, and improvement on related technologies obtained from deep learning. This makes it more suitable for the research topic of this article and design-related experiments and analysis to explore its related performance. The experimental results in this paper show that the improved image recognition technology has improved accuracy by 31.2%. And the performance of its algorithm is also improved by 21%, which can be very effective in monitoring preschool children during breakdancing.

## 1. Introduction

In December 2020, the International Olympic Committee decided to break dancing as an official event of the 2024 Paris Olympics. As early as 2018, at the Youth Olympic Games held in Buenos Aires, Argentina, break dancing appeared beautifully as an official event. The participation of breakdancing in the Olympics, along with the development trend of the times, stimulates new audiences and fascinates young people. This reflects the audiovisual, cultural, and participation nature of the Olympic Games. This greatly increased the social attention of the project and stimulated more children and young people's interest in learning breakdancing. This paper, from the perspective of image recognition technology, combines the neural network of deep learning to carry out a hardcover recognition of the relevant actions in the actual breakdance movement of preschool children, in order to better improve their execution ability.

Break dancing is a comprehensive art form that integrates rhythm, movement, music, and other characteristics. The learning of breakdance requires not only the coordination between individual sensory systems but also the strong coordination between music rhythms and body movements. However, only a few existing studies have explored the impact of breakdancing training on adult emotions, physical value, and interpersonal perception.

The innovation of this article is to take the executive function of preschool children as the theoretical research foundation. And it improves it on the basis of image recognition technology and proposes a neural network image recognition technology based on a deep learning algorithm. This makes it possible to provide more accurate images for the research topic of this article, so as to facilitate the intervention analysis of the executive function of preschool children.

## 2. Related Work

Music, mindfulness, exercise, and other training methods have been used in the study of children's executive ability in the past to promote the development of preschool children's executive function. Although various methods have certain effects, researchers have been exploring more comprehensive methods for effective training. Chui et al. verify that the automatic food image recognition system DietCam (not yet verified) can recognize foods of different shapes and complexity from passively captured digital images. It allows participants to wear Sony smart glasses and automatically take three images per second [1]. Aiming at the problem of low accuracy of the results obtained by traditional methods, Han uses spectral detection in soil pollution component detection methods to design multicolor heavy metal image recognition. He used a spectrometer to measure the soil reflectance spectrum to obtain soil heavy metal spectrum data [2]. Faulkner et al. challenged the computational image analysis of complex subcellular structures with high-throughput confocal imaging. He developed CellArchitect, an automatic image analysis tool that quantifies the changes in the subcellular patterns shown by microtubule markers in plants [3]. Liang et al. proposed a CNN-based multilabel learning model to identify distortions in different scenarios. It includes images without distortion, single distortion, and multiple distortion [4]. Zhang et al. have described an effective metric learning method for the task of identifying flower varieties. It not only provides a high recognition rate but also makes the features extracted from the recognition network interpretable [5]. Aprahamian challenges this narrative by introducing the voices of the founding practitioners that break is often overlooked. By juxtaposing the main testimony with the mainstream performance, his goal is to show how women have played a key role in dance in history and how hegemonic discourse obscured their understanding of the origins of hip hop. He also considered how to reveal the role of women in Break history and reconstruct the popular concept of gender expression [6]. Chen et al. proposed a new method based on Convolutional Neural Network (CNN) to adaptively learn and recognize the discriminative features of typical image processing operations. They carefully designed the high-pass filter bank to obtain the image residual of the input image, the channel expansion layer to mix the result residual, the pooling layer, and the activation function used in their method [7]. Zhang et al. proposed that in recent years, pedestrian reidentification technology has been successfully applied in many fields such as suspect tracking and personnel positioning. Since videos always contain more valuable information, however, most of the existing IVPR models are under the supervision framework. In fact, marking enough training samples requires a lot of manpower, which limits their practical value [8]. The above articles are very detailed about the related image recognition technology and the description of breakdancing. There is also a demonstration of its specific technical key points, but there is no document that combines the two for research and analysis.

## 3. Image Recognition Method Based on Deep Learning

### 3.1. Image Recognition System

In many cases, the information conveyed by images is richer and more realistic than any other form of information [9]. The application of image recognition technology is shown in Figure 1.

Due to the development of digital image technology and the necessity of practicality, other types of problems have occurred [10]. That is, the resulting output does not need to be a complete image. The image after image processing is segmented and effectively extracted: for example, segmentation of various crops, forest resources, mineral resources, and other applications from remote sensing images [11].

Especially with the improvement of the level of science and technology, various research objects can be “imaged” or “digitized.” Using specific technology, the survey object can be converted into images, waveforms, and multiple data. These data can represent all survey subjects. However, in pattern recognition, whether it is data, signal, flat image, or three-dimensional scene, the physical content will be deleted. It finds common points, classifies those with the same common points into one category, and includes other common points. The purpose of image pattern recognition is not humans to complete the task of classification and recognition but to develop and adopt certain machines or machines that automatically process information and perform image recognition quickly and accurately [12]. Generally speaking, an image recognition system consists of the following parts. Its block diagram is shown as in Figure 2.

To build a neural network classifier, it must first choose a suitable network structure. The input of the neural network classifier is the feature vector of the image. The output nodes of the neural network classifier are the number of categories and the number of hidden [13, 14]. It must select a layer and appropriately select the number of neurons in each layer, and there are many network structures that use hidden layers. Next, it must choose an appropriate learning algorithm to obtain a better recognition effect. In the learning phase, training and learning need to use a lot of samples. In addition, multiple samples must be used to correct the weight of the connections of each layer of the neural network. As long as most of the characteristics are consistent with the learned sample, it can be identified as the same category [15].

### 3.2. Deep Learning Methods

Through multilevel feature transformation, another approximate lossless expression is obtained, which is automatic coding [16, 17]. In order to get such an encoder, we usually use the training method shown in Figure 3.

Even if they are not equal, we can adjust the parameters to obtain a reliable encoder. We can cascade multilayer encoders to achieve the output form we want [18]. It adds a classifier behind the cascaded encoder and then uses the supervised training method to train the classifier to get the classification network we want. It is shown in Figure 4.

#### 3.2.1. Sparse Coding

Sparse coding is to express a signal as a linear combination of a set of bases and requires only a few bases to be able to express the signal, as shown in the following formula:

(1) $$\begin{array}{c} x=\overset{k}{\underset{i=1}{\sum }}a_{i}\varphi_{i}, \end{array}$$

where *X* represents the output signal, *φ*_*i*_ represents the base, and *a*_*i*_ is its corresponding coefficient. In order to find a suitable basis and its coefficients, we usually turn it into an optimization problem. It learns and trains the optimal expression by solving Equation (2). Among them, *I* represents the input signal, *O* represents the output signal, and *μ* is the weighting factor.

(2) $$\begin{array}{c} \mathrm{Min}\left(\left(\left|I-\left.0\right|\right.\right)+\mu \times \left(\left|a_{1}\right|+\left|a_{2}\right|+\cdots \left|a_{n}\right|\right)\right). \end{array}$$

#### 3.2.2. Neuron Model

Simply put a neuron node is a nonlinear activation function that receives multiple input values and records it as

(3) $$\begin{array}{c} x=\left(x_{1},x_{2},\cdots x_{n}\right). \end{array}$$

Then, the input signal *X* is weighted and summed to obtain *Z*. Finally, *Z* passes through a nonlinear activation function and outputs the activation value, as shown in the following formula:

(4) $$\begin{array}{c} z=\underset{i=0}{\sum }w_{i}*x_{i}+b,\\ a=f\left(z\right). \end{array}$$

Among them, *W*_*i*_ represents the weight parameter, and *b* is the bias term.

#### 3.2.3. Feedforward Neural Network

Given a group of neurons, we can form a hidden layer or input output layer. It can further connect these layers together to form a network [19]. Neural networks can have many topological structures, and the simplest and most commonly used one is the feedforward neural network.

The data propagation formula of the feedforward neural network is as follows:

(5) $$\begin{array}{c} z^{l}=w^{l}\cdot a^{l-1}+b^{l},\\ a^{l}=f_{l}\left(z^{l}\right). \end{array}$$

Combining the above formulas can be written as

(6) $$\begin{array}{c} z^{l}=W^{l}\cdot f_{l}\left(z^{l-1}\right)+b^{l}. \end{array}$$

According to the above formula, the feedforward neural network passes the input information layer by layer to the next layer, and finally the output of the network is as follows:

(7) $$\begin{array}{c} x=a^{0}⟶z^{1}⟶a^{1}⟶z^{2}⟶\cdots ⟶a^{L-1}⟶z^{L}⟶a^{L}=y. \end{array}$$

#### 3.2.4. Backpropagation Algorithm

Generally, as long as there is large enough dataset and training samples, we can train a neural network with good performance [20]. The objective function is

(8) $$\begin{array}{c} J\left(W,b\right)=\overset{N}{\underset{i=1}{\sum }}L\left(y^{i},f\left(x^{i}\left|W,b\right.\right)\right)+\frac{1}{2}\lambda {\left|\left|W\right|\right|}_{F}^{2},\\ J\left(W,b\right)=\overset{N}{\underset{i=1}{\sum }}J\left(W,b,x^{i},y^{i}\right)+\frac{1}{2}\lambda {\left|\left|W\right|\right|}_{F}^{2}. \end{array}$$

In the above formula, *W* and *b* contain the weight matrix and bias vector of each layer in the network, *λ* is the penalty coefficient of the regular term, and our goal is to minimize it. Here, we can use the stochastic gradient descent method to update the parameters, as follows:

(9) $$\begin{array}{c} W^{l}=W^{l}-\alpha \frac{\partial J\left(W,b\right)}{\partial W^{l}},\\ b^{l}=b^{l}-\alpha \frac{\partial J\left(W,b\right)}{\partial b}, \end{array}$$

where *α* is the learning rate of the parameter.

In order to update, we transform it as follows.

(10) $$\begin{array}{c} \frac{\partial J\left(W,b;x,y\right)}{\partial W_{ij}^{l}}=tr\left({\left(\frac{\partial J\left(W,b;x,y\right)}{\partial z^{l}}\right)}^{T}\frac{\partial z^{l}}{\partial W_{ij}^{l}}\right). \end{array}$$

For the *L*th layer, we define an error term:

(11) $$\begin{array}{c} \delta^{l}=\frac{\partial J\left(W,b;x,y\right)}{\partial z^{l}}\in R^{n^{l}}, \end{array}$$

because

(12) $$\begin{array}{c} z^{l}=W^{l}\cdot a^{l-1}+b^{l}. \end{array}$$

So the following formula can be obtained:

(13) $$\begin{array}{c} \frac{\partial z^{l}}{\partial W_{ij}^{l}}=\frac{\partial \left(W^{l}\cdot a^{l-1}+b^{l}\right)}{\partial W_{ij}^{l}},\\ \frac{\partial z^{l}}{\partial W_{ij}^{l}}=\left[\begin{array}{ccccc} & & 0 & & \\ & & \vdots & & \\ 0 & \cdots & a_{j}^{l-1} & \cdots & 0\\ & & \vdots & & \\ & & 0 & & \end{array}\right]. \end{array}$$

So get

(14) $$\begin{array}{c} \frac{\partial J\left(W,b;x,y\right)}{\partial W_{ij}^{l}}=\delta^{l}a_{j}^{l-1}. \end{array}$$

Further, sort out

(15) $$\begin{array}{c} \frac{\partial J\left(W,b;x,y\right)}{\partial W_{ij}^{l}}=\delta^{l}{\left(a_{j}^{l-1}\right)}^{T}. \end{array}$$

The same can be obtained:

(16) $$\begin{array}{c} \frac{\partial J\left(W,b;x,y\right)}{\partial b^{l}}=\delta^{l}. \end{array}$$

Next, we further solve the error term of the *L*th layer:

(17) $$\begin{array}{c} \delta^{l}\overset{\Delta }{=}\frac{\partial J\left(W,b;x,y\right)}{\partial z^{l}}. \end{array}$$

From the above formula, we can see that after calculating the error term of each layer, we can update the parameters according to the gradient of the parameters of each layer [21]. The training process of the feedforward neural network can be divided into the following three steps:

1. It calculates the state and activation value of each layer according to the forward propagation formula
2. It calculates the error term of each layer according to the back propagation formula
3. It calculates the partial derivative of each layer and updates the parameters

### 3.3. Executive Function of Preschool Children

The concept of executive function originated from Europe and began with the study of patients with frontal lobe damage by British scholars. After the frontal lobe is damaged, the patient can only complete simple tasks but is unable to handle relatively complex tasks. Such tasks usually require corresponding plans and monitoring of completion progress. With the deepening of understanding, researchers believe that executive function is not entirely determined by the function of the prefrontal cortex of the brain but is also related to some other limbic system and cerebral cortex.

Although the division of executive functions by experts and scholars is not consistent, however, by combining various viewpoints and current research trends, it is not difficult to find that the three subfunctions of executive function, inhibitory control, working memory, and cognitive flexibility, have been recognized by most scholars and have been widely used in experimental research. The details are shown in Figure 5.

If inhibition and control are impaired, we will be subjected to impulse, old thinking, or behavioral habits. Therefore, inhibitory control allows us to control our own reactions and behaviors, rather than becoming habitual creatures without thinking. But it is not easy. Our behavior is often controlled by environmental stimuli. But the ability to inhibit control gives us the ability to change and choose, which can help us overcome instinct.

Working memory is different from short-term memory. In addition to remembering information, it also needs to process information. But generally, it cannot handle more than 4 tasks at the same time. Working memory is very important for understanding the context of things, but without working memory, reasoning cannot be carried out. Working memory is vital to our ability to discover connections between seemingly unrelated things, to separate elements from the whole, and to creativity, because creativity involves breaking down and reorganizing elements in new ways. When we read or listen, working memory can help us understand the information received. We cannot do any mathematical calculations without the operation of working memory.

Cognitive flexibility refers to the ability to flexibly switch between tasks, change perspectives or methods, and adjust flexibly to adapt to new changes and rules. Cognitive flexibility can not only change perspectives in space and look at things from different directions but also switch between individuals and look at things from the perspective of others. In this process, we need to suppress the previous angle first and then connect it to the current angle. Cognitive flexibility can also make us jump out of the previous framework and change the way we think about things. It also includes being flexible enough to adapt to changing situations or adjust the priority of tasks. There are many overlaps between cognitive flexibility, task switching, set switching, and creativity, which are rigid opposites. For the impact of breakdancing in this article on the executive function of preschool children, it mainly uses image recognition technology to analyze the actions in breakdancing, so as to better help children improve their executive functions. The recognition action in the process of break dancing is shown in Figure 6.

Executive function is an advanced cognitive function. It has an important influence on children's intellectual development and social behavior. In the early stages of growth, the development of executive function is closely related to children's behavior. Children with poor executive function may have not only learning disabilities but also other behavioral and emotional problems, such as attention deficit hyperactivity disorder, loneliness, depression, and other problems. Meta-analysis has confirmed that older children with disruptive behavior disorders perform poorly in inhibitory tasks.

Executive function measurement is considered to be a novel, complex assessment task involving information integration, and executive function is a complex cognitive process. In the current research, the tests to evaluate the inhibitory control ability of preschool children mainly include flanking tasks, spatial conflict arrow tasks, AnimalGo/NoGotask, delayed gratification tasks, panda/lion, and grass/snow tasks. The tests that assess the working memory ability of preschool children mainly include working memory span tasks, the Coase building block test and the anti-Coase building block test, and the Cambridge neuropsychological test.

As we all know, the level of interest and motivation will affect the performance of cognitive tasks. Young children's motivation and interest levels fluctuate greatly, and they are prone to fatigue, and it is difficult to continue to pay attention during the cognitive assessment process. Therefore, in the evaluation process, in order to improve compliance, a series of measures are often taken. For example, when the child is in good condition, we will arrange multiple tests in a short period of time, and give encouragement to the child at the right time during the experiment. In addition, because preschoolers are now exposed to emerging technologies earlier, if they want to continue to attract this age group, the presentation of many traditional preschool assessment tasks may need to be updated. For example, it can be tested by computers, tablets, game consoles, and other devices. At the same time, the use of these platforms will make the test more objective and can record and save detailed information during the test.

## 4. Intervention Experiment of Break Dance on Executive Function

### 4.1. Executive Function Intervention Experiment

This study took 61 children in a kindergarten class in Dalian as the research object. There were 16 males in the experimental class, 15 males in the control class, 14 females in the experimental class, and 15 females in the control class. One of the classes was randomly selected as the experimental class and the other as the control class (see Table 1 for the mean monthly age and standard deviation).

Adopt 2 × 2 experimental class and control class before and after test design.

This study refers to the requirements and principles of successful promotion of executive function summarized by some experts.

It is divided into four stages: one week in each stage, learning the content of the five levels of breakdancing and the accompaniment is selected from the examination repertoire, including Hook exercises. In this process, the image recognition technology based on deep learning proposed in this paper is used to identify the breakdance movements of preschool children during the practice process and obtain relevant parameters to provide suggestions. The specific training arrangements are shown in Table 2.

Other than this, the daily activities of other kindergartens were consistent. Uniform requirements are imposed on all teachers, and teachers cannot impose additional activities on preschool children.

In the homogeneity test of the children in the experimental class and the control class before breakdancing training (as shown in Table 3), the test results show that there is no difference in the executive function level of the children in the experimental class and the control class in the pretest (*t*-test is not significant).

This experiment is an educational field experiment and is a quasiexperimental design. During the demonstration phase, place the two sorting trays side by side in front of the subject, ensuring that they are within reaching distance. Sit beside the child so that you are able to view the display panels. Affix target cards to the display panels behind the sorting trays (e.g., a blue rabbit behind the tray on the child's left and a red boat behind the tray on the child's right). Label the target cards by both dimensions. Say, “Here's a blue rabbit and here's a red boat.” Then say, “Now, we are going to play a card game.” The result is shown in Figure 7.

A two-factor repeated measurement analysis of variance of 2 (pre‐and posttest) × 2 (class type) is done. Among them, the before and after measurements are variables within the group, and the class type is the variable between groups. The analysis of variance mainly examines the interaction between pre- and posttest and class type (as shown in Tables 4 and 5). The specific results are as follows:

The results show that the 8-week breakdancing training can promote the development of executive function of preschool children.

In the past, breakdancing training mostly used teenagers or college students as the training objects to explore the impact of breakdancing training on their physical and mental health. It is conducive to the development of physical and mental health of preschool children and the improvement of living standards.

In order to better obtain the recognition ability of the algorithm proposed in this paper for breakdance movements and in order to better promote the executive function of preschool children, this paper designs the algorithm ability analysis part to recognize the action of the algorithm in different aspects: ability and other related factors, to carry out research analysis to compare the superiority of the algorithm.

## 5. Algorithm Ability

### 5.1. The Correct Rate under Different Pruning Ratios

In order to compress the size of the CNN model as much as possible and find the appropriate pruning ratio, we conducted multiple experiments on the pruning ratio. Because the parameter scale of the fully connected layer is the largest, it can account for more than 90% of the parameter scale of the entire model. So we first experimented on the pruning ratio of the fully connected layer and then compared the pruning ratio of the first five convolutional layers. The experimental results are shown in Figure 8.

Through model pruning, not only the scale of the model is reduced but also the amount of calculation in the forward propagation process of the network is greatly reduced. Compared with the nonpruned network model, the network model after pruning has only 30% of the original calculation amount, which increases the detection speed of the algorithm network by 3 times and greatly improves the performance of the algorithm.

### 5.2. Action Recognition Analysis

In order to evaluate the effectiveness of the proposed method, experimental analysis was carried out on three public mainstream breakdancing action databases. The video gradually expands from neutral action to one of seven kinds of actions, and the maximum action intensity of the last frame is the peak frame of the entire video. The training loss and accuracy of the validation set are shown in Figure 9.

The training loss represents the data lost in the process of training the actual dataset, and the verification accuracy is the probability of being able to study correctly. The database includes 213 frontal image sequences from 31 people. Each of its videos contains the complete process of action expression and restoration; that is, it gradually develops from a neutral action to one of the six basic actions over time and then gradually releases the action and returns to the neutral action. It can be seen that the method proposed in this paper effectively exceeds the previous algorithm.

#### 5.2.1. Test Results Based on the IJB-A/B/C Dataset

The IJB-A dataset is an image set captured in an unconstrained environment, and its pose and imaging conditions vary greatly. It was collected from 500 individuals, with a total of 25,813 images. There are 10 training and test divisions for 10-fold cross-validation. Each fold contains 333 training and 167 test identities, and the test results are shown in Figure 10.

These results show that, compared with the original method, the verification and identification performance of the method proposed in this paper have been greatly improved. It shows that this method is obviously better than the previous method and can better stabilize its effect in training.

### 5.3. Test Results Based on the Celebrity-1000 Dataset

Finally, the method proposed in this paper is tested on the Celebrity-1000 dataset, which is designed for unconstrained video-based action recognition problems. This dataset contains 2.4 million frames from 159,726 facial action videos, including 1,000 individuals. It has two standard test procedures, namely, open set and closed set. Follow the standard 1 : N discrimination setting, and report the results of the two tests. The results are shown in Figure 11.

In the three experiments, the performance comparison is shown from the perspective of deep reinforcement learning. For a good learning algorithm, there is a higher reward. For the challenging poses in the collection and action recognition datasets, the action and imaging conditions are relatively robust.

### 5.4. Analysis

Based on the above analysis, it is not difficult to see that the improved image recognition based on neural network learning can more accurately intervene in the executive function of preschool children. The accuracy of the improved image recognition has increased by 31.2%, and the algorithm performance has increased by 21%. This is a huge improvement in the ability of image recognition and can be better applied to breakdancing interventions in the executive function of preschool children.

## 6. Conclusions

This article is mainly to carry out a promotion intervention on the executive function of preschool children under the breakdancing sport. Through the use of image recognition algorithms, children's breakdancing work can be better captured, so as to study the actions of preschool children and analyze the improvement of their executive functions. This paper proposes a neural network image recognition technology based on deep learning and improves the learning method of deep learning, which makes the improved learning ability stronger and more suitable for the research topic of this paper. And the key algorithm is improved, and it is improved to the neural network image recognition based on deep learning, so that it can be better applied to the research topic of this article. Finally, a related experiment was designed to investigate the breakdancing of preschool children, and the performance of the algorithm was studied in the analysis part to ensure the stable operation of the algorithm. At the same time, in the future, for the combination of image recognition technology and neural network, it is also necessary to use more data sets to recognize and train it, so that it can be more accurate in the actual action recognition process.

## Figures and Tables

**Figure 1:** Application of image recognition technology.

**Figure 2:** Block diagram of image recognition system.

**Figure 3:** Structure diagram of training autoencoder.

**Figure 4:** Structure diagram of training cascade encoder classification.

**Figure 5:** Subfunction division of executive functions.

**Figure 6:** Breakdancing action based on image recognition.

**Figure 7:** The flow of the presentation phase.

**Figure 8:** The accuracy of the three fully connected layers under different pruning ratios.

**Figure 9:** Comparison of training loss and accuracy of validation set before and after improvement.

**Figure 10:** Comparison of average ROC curve and CMC curve.

**Figure 11:** Performance comparison on three datasets.

**Table 1:** Basic situation of the subjects.

Grouping	Experimental class	Control class
Total number of participants	30 pieces	31 pieces
Male	16 pieces	15 pieces
Female	14 pieces	16 pieces
Average age	59.47	59.12
Standard deviation	1.77	1.94

**Table 2:** “Five Levels of Street Dance” training plan.

Week	Training category	Item number	Training content	Training goal
3	Hook	12	Squat balance	Cognitive flexibility
		13	Hand changes	Working memory
		14	Hip swing	Inhibition control
		15	Hook exercise	Inhibition control

**Table 3:** Homogeneity test before experiment.

Test content	Experimental class	Control class	*t*
Stroop test	12.83	11.86	0.674
Dimension change card sort	12.45	12.59	-1.14
Points memory task	0.84	0.74	1.278
Reverse counting task	7.34	6.51	0.246

**Table 4:** The average score and standard deviation of each component of the executive function of the experimental class and the control class.

Test content	Experimental class		Control class	
	Pretest	Posttest	Pretest	Posttest
Stroop test	12.81 ± 4.51	23.17 ± 1.18	11.85 ± 6.28	17.56 ± 4.64
Dimension change card sort	12.41 ± 2.84	15.63 ± 1.81	12.51 ± 2.84	13.59 ± 2.34
Points memory task	7.31 ± 2.14	8.78 ± 1.78	6.52 ± 2.31	6.94 ± 1.98
Reverse counting task	0.84 ± 0.869	1.82 ± 0.754	0.76 ± 0.86	0.84 ± 0.86

**Table 5:** Analysis of variance of two-factor mixed experimental design.

Test content	Source	df	MS	*F*	*η* ^2^ *ρ*
Stroop task	Time	1	2187.549	141.759	0.714
	Between groups	1	227.189	9.024	0.126
	Time∗between groups	1	97.214	6.328	0.089
	Time	1	127.354	27.498	0.318

## Data Availability

The experimental data used to support the findings of this study are available from the corresponding author upon request.
